This article has been retracted.

# Bone Marrow Mesenchymal Stem Cell-Derived Exosomal MicroRNA-126-3p Inhibits Pancreatic Cancer Development by Targeting ADAM9

**DOI:** 10.1016/j.omtn.2019.02.022

**Published:** 2019-03-01

**Authors:** Dong-Mei Wu, Xin Wen, Xin-Rui Han, Shan Wang, Yong-Jian Wang, Min Shen, Shao-Hua Fan, Zi-Feng Zhang, Qun Shan, Meng-Qiu Li, Bin Hu, Jun Lu, Gui-Quan Chen, Yuan-Lin Zheng

**Affiliations:** 1 Key Laboratory for Biotechnology on Medicinal Plants of Jiangsu Province, School of Life Science, Jiangsu Normal University, Xuzhou 221116, China; 2 College of Health Sciences, Jiangsu Normal University, Xuzhou 221116, Jiangsu, China; 3 State Key Laboratory of Pharmaceutical Biotechnology, MOE Key Laboratory of Model Animal for Disease Study, Model Animal Research Center, Nanjing University, Nanjing 210061, Jiangsu, China

**Keywords:** bone marrow mesenchymal stem cells, exosomes, microRNA-126-3p, a disintegrin and a metalloproteinase-9, pancreatic cancer, invasion, metastasis

## Abstract

Pancreatic cancer is a lethal malignancy with relatively few effective therapies. Recent investigations have highlighted the role of microRNAs (miRNAs) as crucial regulators in various tumor processes including tumor progression. Hence the current study aimed to investigate the role of bone marrow mesenchymal stem cell (BMSC)-derived exosomal microRNA-126-3p (miR-126-3p) in pancreatic cancer. Initially, miRNA candidates and related genes associated with pancreatic cancer were screened. PANC-1 cells were transfected with miR-126-3p or silenced a disintegrin and a metalloproteinase-9 (ADAM9) to examine their regulatory roles in pancreatic cancer cells. Additionally, exosomes derived from BMSCs were isolated and co-cultured with pancreatic cancer cells to elucidate the effects of exosomes in pancreatic cancer. Furthermore, the effects of overexpressed miR-126-3p derived from BMSCs exosomes on proliferation, migration, invasion, apoptosis, tumor growth, and metastasis of pancreatic cancer cells were analyzed in connection with lentiviral packaged miR-126-3p *in vivo*. Restored miR-126-3p was observed to suppress pancreatic cancer through downregulating ADAM9. Notably, overexpressed miR-126-3p derived from BMSCs exosomes inhibited the proliferation, invasion, and metastasis of pancreatic cancer cells, and promoted their apoptosis both *in vitro* and *in vivo*. Taken together, the key findings of the study indicated that overexpressed miR-126-3p derived from BMSCs exosomes inhibited the development of pancreatic cancer through the downregulation of ADAM9, highlighting the potential of miR-126-3p as a novel biomarker for pancreatic cancer treatment.

## Introduction

Pancreatic cancer is a major threat to human health with very few effective therapies and prognoses.^1^, ^2^, ^3^ As the fourth primary death cause of all different cancers, the survival rate of pancreatic cancer is incredibly low.^4^ Despite improvements made to pancreatic cancer therapies, the mortality of the disease has remained more or less the same over the past several decades, largely due to the lack of adequate screening methods and biomarkers for early diagnosis.^5^ Four decades ago, bone marrow mesenchymal stem cells (BMSCs) were found in bone and cartilage comprised of approximately 0.001%–0.01% of the marrow nuclear cells. BMSCs can be defined as a family of non-hematopoietic cells similar to fibroblast and first used as multipotent progenitor cells.^6^, ^7^ That being said, reports have suggested that BMSCs could promote the development of cancer,^8^, ^9^, ^10^ while existing literature has emphasized the potential of BMSCs from a therapeutic perspective for patients suffering from amyotrophic lateral sclerosis due to its safety and effectiveness.^11^ Remarkably, BMSCs have been shown to be capable of migrating to tumor tissues, while studies have speculated their potential for gene therapy in cases of pancreatic cancer.^12^

Exosomes are small, membrane-enclosed vesicles (30–150 nm) that can deliver cargo (proteins, lipids, and nucleic acids) from the originating cells to the recipient cells.^13^ Recently, a type of small vesicle released from marrow mesenchymal stem cell (MSC)-derived exosomes has been shown to transfer functional RNAs to recipient cells, indicating their promise as an alternative for cell-based therapy.^14^ Especially, it was reported that exosomes could carry microRNAs (miRNAs), which are involved in cancer cell proliferation, differentiation, and apoptosis.^15^, ^16^ Moreover, as tumor suppressors or oncogenes, miRNAs regulate gene expression post-transcriptionally.^17^ For instance, miR-126-3p, a subtype miRNA, has been shown to act as a tumor suppressor, while reports have suggested that it may be capable of suppressing the progression of cancer.^18^, ^19^ Besides, miR-126-3p has been found to exhibit downregulated levels in esophageal squamous cell carcinoma (ESCC), especially in cases with poor prognosis.^20^ Additionally, miR-126-3p has been reported to be capable of inhibiting cellular metastasis, invasion, and dysregulation within the plasm of pancreatic cancer patients.^21^ Based on the exploration of literature, it was asserted that miR-126-3p could serve as a therapeutic target. Interestingly, miR-126-3p was previously reported to negatively regulate a disintegrin and a metalloproteinase-9 (ADAM9).^22^ ADAM9 is a type I membrane-anchored protein that has been correlated with the development of cancers because of its high expression levels in metastatic cancer.^23^ Growing evidence continues to suggest that the miR-126/ADAM9 axis could suppress the progression of pancreatic cells.^24^ Hence the hypothesis was asserted that overexpressed miR-126-3p derived from BMSCs exosomes could suppress the progression of pancreatic cancer via the downregulation of ADAM9. Hence the aim of the current study was to explore the effects of miR-126-3p transferred by BMSC-derived exosomes in pancreatic cancer.

## Results

### miR-126 Targets ADAM9 in Pancreatic Cancer

Initially, R language was employed to screen for differentially expressed genes from four gene expression chips of pancreatic cancer (GEO: GSE16515, GSE32676, GSE71989, and GSE101448) with |log2 fold change (FC)| > 1.0 and *adj.P.Val* < 0.05 set as the screening threshold. The first 400 differentially expressed genes of each chip were compared and plotted in Venn diagram. As illustrated in Figure 1A, ADAM9 was determined to be the exclusive intersection gene. The detailed results of the initial 400 differentially expressed genes of each chip are depicted in Table S1. The expression of the thermal map of the first 60 differentially expressed genes from the GEO: GSE101448 and GSE32676 chips were plotted, respectively (Figures 1B and 1C). The expression of ADAM9 in pancreatic cancer tissues was found to be higher than that of the normal tissues. Similarly, our results revealed that ADAM9 was highly expressed in the pancreatic cancer tissues from the GEO: GSE16515 and GSE71989 chips when compared with the normal tissue (Figures 1D and 1E). In order to verify the expression of ADAM9 and analyze the correlation between gene expression and survival conditions, the Gene Expression Profiling Interactive Analysis (GEPIA) database was explored to determine and retrieve the expression of ADAM9 in both pancreatic cancer tissues and normal tissues. The expression of ADAM9 in the pancreatic cancer tissues was higher than normal tissues (Figure 1F). Notably, the survival analysis (Figure 1G) revealed that the higher the expression of ADAM9, the lower the total survival rate of patients with pancreatic cancer.

**Figure 1:** ADAM9 Was the Target of miR-126 (A) The first 400 differentially expressed genes of pancreatic cancer gene expression chips (GEO: GSE16515, GSE32676, GSE71989, and GSE101448), with one intersection gene ADAM9 observed. (B and C) Thermal map of the first 60 genes of the gene expression chips GEO: GSE101448 (B) and GSE32676 (C), respectively. The abscissa was representative of the sample number, whereas the ordinate was reflective of the differentially expressed genes. The upper right histogram is the color order, and each rectangle in the graph corresponds to a sample expression value. (D and E) The expression of ADAM9 in (D) GEO: GSE16515 and (E) GSE71989 gene chips, respectively. (F) The expression of ADAM9 in pancreatic cancer tissues and normal tissues retrieved from the GEPIA database. *p < 0.01. (G) The correlation between ADAM9 expression and total survival rate in patients with pancreatic cancer in the GEPIA database. (H) The comparison of target miRNA of ADAM9 predicted by TargetScan, miRSearch, miRTarBase, miRWalk, and mirDIP. (I) The expression of hsa-miR-126-3p in miRNA expression chip GEO: GSE28955 of pancreatic cancer. ADAM9, a disintegrin and a metalloproteinase-9; GEPIA, Gene Expression Profiling Interactive Analysis; miR-126, microRNA-126.

To further predict the miRNA regulating ADAM9, five miRNA-mRNA relation prediction databases (TargetScan, miRSearch, miRTarBase, miRWalk, and mirDIP) were used to predict the target miRNA, after which the results obtained were compared with the predicted results. The detailed results are displayed in Table S2. In accordance with the Venn diagram (Figure 1H), three intersection miRNAs, hsa-miR-26b-5p, hsa-miR-126-3p, and hsa-miR-373-3p, were found by comparison of five miRNA prediction results, indicating that these three miRNAs were highly likely to regulate ADAM9. Furthermore, through screening of the miRNA expression chip GEO: GSE28955 of pancreatic cancer by R, among the three aforementioned miRNAs that targeted ADAM9, only hsa-miR-126-3p was poorly expressed in pancreatic cancer tissues (Figure 1I), suggesting that miR-126 could target ADAM9 in pancreatic cancer. The specific expression data of ADAM9 and hsa-miR-126 are depicted in Table S3.

### miR-126-3p Is Poorly Expressed in Pancreatic Cancer Cells

In order to ascertain whether the expression of miR-126-3p is altered in pancreatic cancer cells, its expression in 28 patients with pancreatic cancer, as well as among 32 patients with pancreatitis, was determined through the application of qRT-PCR. The expression of miR-126-3p in the pancreatic cancer tissues was markedly lower than the results of the patients with pancreatitis (Figure 2A), suggesting that miR-126-3p is downregulated in pancreatic cancer cells. In addition, qRT-PCR was employed to detect the expression of miR-126-3p in the normal human pancreatic cell line HPC-Y5, with six pancreatic cancer cell lines (PANC-1, SW1990, Capan-1, AsPC-1, PC-3, and MIAPaCa-2 cell lines) screened in order to detect the cell line with the poorest expression of miR-126-3p. The results obtained distinctly indicated that the expression of miR-126-3p was decreased among all the pancreatic cancer cell lines when compared with the normal pancreatic cell line HPC-Y5 (Figure 2B), with the expression of miR-126-3p in PANC-1 found to be the lowest (p < 0.05) among all tested pancreatic cancer cell lines. Thus, PANC-1 was selected for subsequent cell experiments.

**Figure 2:** Pancreatic Cancer Tissues Exhibited Reduced Expression of miR-126-3p (A) The relative expression of miR-126-3p in pancreatic cancer tissues and pancreatitis tissues (pancreatic cancer: n = 28, pancreatitis: n = 32) (*p < 0.05, compared with the normal group). (B) Relative expression of miR-126-3p in human normal pancreatic cell line HPC-Y5 and six pancreatic cancer cell lines detected by qRT-PCR (*p < 0.05, compared with HPC-Y5). The measurement data were expressed as mean ± SD. The data are between two groups compared with the independent sample t test. Data among multiple groups were compared using one-way ANOVA. The experiment was repeated three times. miR-126-3p, microRNA-126-3p.

### miR-126-3p Inhibits Proliferation, Migration, and Invasion of Pancreatic Cancer Cells and Promotes Their Apoptosis

In order to examine the influence of miR-126-3p on pancreatic cancer cells, PANC-1 was treated with a mimic and inhibitor of miR-126-3p. The results (Figures 3A–3D) revealed that when compared with the mimic-negative control (NC) group, the cell proliferation, migration, and invasion abilities were decreased, whereas the apoptotic rate was elevated in the miR-126-3p mimic group (p < 0.05). In contrast, when compared with the inhibitor-NC group, the miR-126-3p inhibitor group exhibited increased cell proliferation, migration, and invasion abilities along with a diminished rate of apoptosis (p < 0.05). Restored miR-126-3p was associated with inhibited proliferation, migration, and invasion of pancreatic cancer cells in addition to stimulated rates of apoptosis, whereas a contradictory trend was observed when miR-126-3p was silenced and opposite outcomes to the above mentioned were exhibited.

**Figure 3:** Overexpressed miR-126-3p Contributed to Inhibited Proliferation, Migration, and Invasion of Pancreatic Cancer Cells and Promoted Their Apoptosis (A) The effect of miR-126-3p on the proliferation of pancreatic cancer cell line PANC-1 detected by EdU assay (original magnification ×400). (B) The effect of miR-126-3p on migration ability of PANC-1 detected by Transwell assay (original magnification ×200). (C) The effect of miR-126-3p on the invasion of PANC-1 detected by Transwell assay (original magnification ×200). (D) The effect of miR-126-3p on the apoptosis rate of PANC-1 detected by flow cytometry. The data in the chart were all measured and expressed as mean ± SD. The independent samples t test was used for statistical analysis between two groups, and the experiment was repeated three times. EdU, 5-ethynyl-2′-deoxyuridine; miR-126-3p, microRNA-126-3p; NC, negative control.

### miR-126-3p Targets ADAM9

Based on the online software analysis, miR-126-3p was detected to have a specific binding region for ADAM9 within its 3′ UTR (Figure 4A). In order to ascertain as to whether miR-126-3p regulates ADAM9 by binding to the predicted target site in the 3′ UTR, a dual-luciferase reporter gene assay was performed (Figure 4B). Compared with the NC group, overexpression of miR-126-3p inhibited the luciferase activity of 3′ UTR of ADAM9-wild-type (WT) (p < 0.05). However, miR-126-3p was found to have no significant effect on the luciferase activity of 3′ UTR ADAM9 mutant (MUT) (p > 0.05), indicating that ADAM9 is a target of miR-126-3p.

**Figure 4:** ADAM9 Was a Direct Target Gene of miR-126-3p (A) The targeting relationship between miR-126-3p and ADAM9 predicted in the biological prediction website microRNA.org (http://www.microrna.org/microrna/home.do). (B) The target relationship between miR-126-3p and ADAM9 verified by dual-luciferase reporter gene assay. (C) mRNA expression of ADAM9 in each group determined by qRT-PCR. (D) Protein expression of ADAM9 in each group measured using western blot analysis. *p < 0.05, compared with the ADAM9-mut group. The data were measured and expressed as mean ± SD. Independent sample t test was used for statistical analysis, and the experiment was repeated three times. ADAM9, a disintegrin and metalloprotease-9; GAPDH, glyceraldehyde-3-phosphate dehydrogenase; miR-126-3p, microRNA-126-3p; MUT, mutant; NC, negative control; WT, wild-type.

qRT-PCR and western blot analysis were then employed to determine the mRNA and protein expression of ADAM9 (Figures 4C and 4D). The expression of ADAM9 gene was decreased when miR-126-3p was overexpressed, while increased levels were noted in the presence of inhibited miR-126-3p (p < 0.05). Accordingly, ADAM9 was the target of miR-126-3p, whereas overexpressed miR-126-3p was observed to downregulate ADAM9 expression.

### miR-126-3p Inhibits Proliferation, Migration, and Invasion of Pancreatic Cancer Cells and Promotes Their Apoptosis by Negatively Regulating ADAM9

ADAM9 was interfered with in order to investigate the molecular mechanisms that underlie the miR-126-3p-mediated inhibition on proliferation, apoptosis, migration, and invasion abilities of pancreatic cancer cells. The results demonstrated (Figures 5A–5D) that compared with the RNA interference of NC (si-NC) group, the cell proliferation, migration, and invasion ability of the si-ADAM9 group were decreased, whereas the apoptotic rate was boosted (p < 0.05). In contrast, compared with the miR-126-3p inhibitor + si-NC group, the proliferation, migration, and invasion ability were reduced, whereas the rate of apoptosis was diminished in the miR-126-3p inhibitor + si-ADAM9 group (p < 0.05). The results of RT-PCR and western blot analysis indicated that the mRNA and protein expression of ADAM9 were decreased (p < 0.05) when compared with the corresponding NC group (Figures 5E and 5F). Taken together, miR-126-3p was ultimately confirmed to inhibit the proliferation, migration, as well as the invasion of pancreatic cancer cells while promoting their apoptosis by negatively regulating ADAM9.

**Figure 5:** miR-126-3p Inhibited Biological Function in Pancreatic Cancer Cells by Negatively Regulating ADAM9 (A) The effect of ADAM9 on the proliferation of PANC-1 detected by EDU assay (original magnification ×400). (B) The effect of ADAM9 on migration ability of PANC-1 using Transwell assay (original magnification ×200). (C) The effect of ADAM9 on the invasiveness of PANC-1 using Transwell assay (original magnification ×200). (D) The effect of ADAM9 on the apoptosis rate of PANC-1 determined by flow cytometry. (E–G) The mRNA and protein expression of ADAM9 gene measured using qRT-PCR (E) and western blot analysis (F and G), respectively. The data were all measured and expressed by mean ± SD. The independent sample t test was used for statistical analysis between two groups, and the experiment was repeated three times. ADAM9, a disintegrin and metalloprotease-9; EdU, 5-ethynyl-2′-deoxyuridine; GAPDH, glyceraldehyde-3-phosphate dehydrogenase; miR-126-3p, microRNA-126-3p; NC, negative control.

### BMSCs Sorting

After the subculture of BMSCs, the aging cells and a small number of mixed cells were eliminated in a progressive fashion. After three to four generations, relatively homogeneous and vigorous purified cells in shuttle shape along with a swirling arrangement were observed (Figures 6A and 6B). The third-generation cells exhibiting good growth were incubated with fluorescein isothiocyanate (FITC)-labeled mouse anti-human antibodies (CD29, CD34, CD44, CD45, CD71, and histocompatibility leukocyte antigen [HLA]-DR) for identification of surface antigen using flow cytometry. Generally, CD29, CD44, and CD71 are considered to be markers of BMSC expression,^25^ CD34 and CD45 are regarded as hematopoietic stem cell markers,^26^ whereas HLA-DR is predominately expressed in certain antigen-presenting cells, such as B lymphocyte, macrophage, and activated T lymphocyte.^27^ CD29 (97.60%), CD44 (98.90%), and CD71 (99%) were found to be positive, whereas HLA-DR (6.11%), CD34 (3.12%), and CD45 (2.41%) were all negative (Figure 6C), supporting that the cultured cells were BMSCs. When cell confluence reached 100%, the BMSCs were cultured with specific culture medium for adipogenic differentiation purposes. Next, 72 h postculture, small lipid droplets were observed in the cells. After culturing for an additional 2 h, a large amount of lipid droplets appeared in the cells in addition to the appearance of a long spindle or polygonal shape. The oil red O staining provided verification indicating that lipid composition was deposited, highlighting the BMSC ability of lipid differentiation (Figure 6D). Following the addition of a specific culture inducing liquid, the BMSCs were differentiated into osteoblasts. After 3 days of induction culture, the cells were in short spindle shape with increased volume. On the seventh day of culture, the cells were observed to have a polygonal shape with calcium granules in the cytoplasm. On the 14th day of culture, the whole cells were filled with calcium granules, and the cells grew in a colony-like manner. The cells at the center were observed to gradually fuse in addition to the loss of their typical cell structure with the formation of clear calcium nodules. The cells were stained red using alizarin red staining and stained black using Von Kossa staining (Figure 6E).

**Figure 6:** Results of BMSCs Sorting (A) Morphology of BMSCs in primary adherent culture (original magnification ×100). (B) The morphology of the third generation BMSCs observed under a microscope (original magnification ×200). (C) Positive markers (CD29, CD44, and CD71) and negative markers (HLA-DR, CD34, and CD45) of BMSCs identified by flow cytometry. (D) Results of oil red O staining after 2 weeks of lipid-induced differentiation (original magnification ×400). (E) Results of alizarin red and Von Kossa staining after 4 weeks of osteogenic induction (original magnification ×400). The data were all measured and expressed by mean ± SD. The independent sample t test was used for statistical analysis between two groups, and the experiment was repeated three times. BMSC, human bone mesenchymal stem cell.

### BMSC-Derived Exosomes Carry miR-126-3p

In order to isolate and subsequently identify the BMSC-derived exosomes, exosomes with the diameter of 60–160 nm were collected by means of ultracentrifugation, exhibiting circular or oval shape with complete membrane structure and low-density substance under transmission electron microscopy (TEM) (Figure 7A). Moreover, in order to determine their respective size distribution, the NanoSightNS300 nanoparticle tracking analysis tool was used. As illustrated in Figure 7B, exosome particles were located predominately around 100 nm. Western blot analysis results revealed that the exosome surface marker proteins CD63 and Hsp70 were specifically detected in BMSC-derived exosomes (Figure 7C). Cy3-labeled exosomes in BMSCs were co-cultured with PANC-1 cell and tagged with GFP for 6 h. Under the confocal fluorescence microscope, slight red fluorescence of Cy3-exosomes could be observed in the PANC-1 cells (Figure 7D), which was indicative of the entrance of a small number of Cy3-exosomes into PANC-1 cells. After a 12-h period of co-culturing, a small number of PANC-1 cells was observed to have exhibited red fluorescence, with the fluorescence mainly concentrated in the cytoplasm, indicating that Cy3-exosomes were mainly located in the cytoplasm of PANC-1 cells. With the prolongation of co-culture time, more PANC-1 cells exhibited red fluorescence, indicating that the number of Cy3-exosomes absorbed by PANC-1 cells increased gradually. At 48 h of co-culture, Cy3-exosomes were obviously absorbed by PANC-1 cells. Notably, the expression of miR-126-3p was found to be markedly higher in the BMSCs, exosomes, and co-cultured pancreatic cancer cells when compared with the NC group (Figure 7E), which suggested that miR-126-3p could be carried by BMSC-derived exosomes. The levels of ADAM9 were further detected and the results demonstrated there to be diminished levels of ADAM9 after the pancreatic cancer cells had absorbed the exosomal miR-126-3p (Figures 7F–7H).

**Figure 7:** miR-126-3p Could Be Carried by BMSC-Derived Exosomes (A) The ultrastructure of exosomes observed by TEM (original magnification ×400). (B) Size distribution of exosomes detected by NanoSight particle size analysis. (C) Surface markers of exosomes (CD63, Hsp70) detected by western blot analysis. (D) The exosomes absorbed by PANC-1 cells under confocal fluorescence microscope at different time points. Red: miR-126-Cy3; green: pCDNA3.1-GFP; blue; DAPI. (E) The expression of miR-126-3p in BMSCs, exosomes, and co-cultured pancreatic cancer cells determined by qRT-PCR. (F) mRNA expression of ADAM9 in pancreatic cancer cells determined by qRT-PCR. (G and H) Protein expression of ADAM9 in pancreatic cancer cells determined by western blot analysis. The data in the chart were analyzed using an independent sample t test, and the experiment was repeated three times. *p < 0.5. BMSC, bone marrow mesenchymal stem cell; GAPDH, glyceraldehyde-3-phosphate dehydrogenase; miR-126-3p, microRNA-126-3p; NC, negative control; TEM, transmission electron microscopy.

### GW4869 Inhibits the Release of BMSC-Derived Exosomes, Thus Suppressing miR-126-3p Expression

In order to further investigate whether miR-126-3p carried by exosomes influences the biological functions of pancreatic cancer cells, the exosomes’ secretory-specific inhibitor GW4869 was added to the co-culture system in the Transwell chamber to elucidate the effect of GW4869 on release of exosomes and the expression of miR-126-3p in pancreatic cancer cells. Compared with the NC DMSO group, the activity of acetylcholinesterase (AChE) in the GW4869 group was decreased, suggesting that the release of the exosomes and the miR-126-3p expression in the exosomes were reduced (p < 0.05; Figures 8A and 8B). Furthermore, the migration and invasion ability of pancreatic cancer cells was higher in the GW4869 group when compared with that of the DMSO group (p < 0.05; Figures 8C–8F). Based on the aforementioned results, it was concluded that GW4869 inhibited the release of BMSC-derived exosomes, resulting in the suppression of miR-126-3p expression.

**Figure 8:** GW4869 Inhibited the Release of BMSC-Derived Exosomes to Inhibit the Expression of miR-126-3p (A) The effect of GW4869 on the release of exosomes detected by AChE activity assay. (B) The effect of GW4869 on the expression of miR-126-3p in pancreatic cancer cells determined using qRT-PCR. (C and E) The effect of GW4869 on migration ability of PANC-1 detected by Transwell assay (photograph of migration cell, C, and number of migration cell, E). (D and F) The effect of GW4869 on invasion of PANC-1 determined by Transwell assay (photograph of invasion cell, D, and number of migration cell, F). The data were measured by the mean ± SD. Comparison between two groups was conducted using an independent sample t test for statistical analysis; *p < 0.05, compared with the DMSO group. The experiment was repeated three times. miR-126-3p, microRNA-126-3p.

### miR-126-3p Transferred by BMSC-Derived Exosomes Suppresses Proliferation, Migration, and Invasion of Pancreatic Cancer Cells and Enhances Their Apoptosis

In order to examine the effect of miR-126-3p in BMSC-derived exosomes on the biological function of pancreatic cancer cells, the cell proliferation, migration, and invasion abilities of pancreatic cancer cells were examined in BMSC-derived exosomes overexpressing miR-126-3p. The results obtained indicated that (Figures 9A–9D), in comparison with the BMSCs-miR-126-3p NC group, the cell proliferation, migration, and invasion abilities of the BMSCs-miR-126-3p mimic group were markedly elevated, whereas the apoptosis rate was notably increased (p < 0.05). Western blot analysis revealed that the expression of proliferation-related factors [Ki67 and vascular endothelial growth factor (VEGF)] and invasive factors [cyclooxygenase-2 (COX-2) and matrix metalloproteinase-14 (MMP-14)] in the BMSCs-miR-126-3p mimic group was significantly lower than that in the BMSCs-miR-126-3p NC group (all p < 0.05; Figures 9E and 9F). The obtained data suggested that BMSCs deliver miR-126-3p via exosomes to inhibit proliferation, migration, and invasion of pancreatic cancer cells and promote their apoptosis.

**Figure 9:** BMSC-Derived Exosomes Transferred miR-126-3p to Pancreatic Cancer Cells to Influence Their Biological Functions (A) Proliferation ability of PANC-1 after transfection detected by EdU assay (original magnification ×400). (B) Apoptosis rate of PANC-1 after transfection determined by flow cytometry. (C) Migration ability of PANC-1 after transfection detected by Transwell assay (original magnification ×200). (D) Invasive ability of PANC-1 after transfection detected by Transwell assay (original magnification ×200). (E) The expression of cell proliferation factor (Ki67 and VEGF) and invasion factor (COX-2 and MMP-14) determined by western blot analysis. (F) Statistical analysis of western blot analysis. The data were measured by the mean ± SD, and the data between two groups were compared with the independent sample t test for statistical analysis. *p < 0.05, compared with the Exo-miR-NC group, and the experiment was repeated three times. BMSC, human bone mesenchymal stem cell; COX-2, cyclooxygenase-2; EdU, 5-ethynyl-2′-deoxyuridine; GAPDH, glyceraldehyde-3-phosphate dehydrogenase; miR-126-3p, microRNA-126-3p; NC, negative control; VEGF, vascular endothelial growth factor.

### miR-126-3p in BMSC-Derived Exosomes Inhibits Tumor Growth and Metastasis of Pancreatic Cancer Cells

In order to investigate the effect of miR-126-3p on tumor growth, overexpressed miR-126-3p in BMSCs was examined by xenograft in nude mice. In contrast with the BMSCs-miR-126-3p NC group, the tumor formation time was shorter, along with a slower growth rate, as well as smaller tumors, in the BMSCs-miR-126-3p mimic group (p < 0.05; Figures 10A–10C). The expression of miR-126-3p and ADAM9 was verified through the application of qRT-PCR and western blot analysis methods, respectively. Compared with the BMSCs-miR-126-3p NC group, the expression of miR-126-3p in the BMSCs-miR-126-3p mimic group was increased significantly (p < 0.05; Figure 10D), whereas that of ADAM9 decreased in a dramatic fashion (p < 0.05; Figure 10D–10F). The expression of COX-2 and MMP-14 in the BMSCs-miR-126-3p mimic group was decreased when compared with the BMSCs-miR-126-3p NC group (p < 0.05; Figure 10D). The results obtained demonstrated that the miR-126-3p expression in the BMSCs-miR-126-3p mimic group was markedly elevated (p < 0.05; Figures 10E and 10F). Taken together, the results obtained suggested that BMSC-derived exosomes transferred miR-126-3p to inhibit proliferation, invasion, and metastasis of pancreatic cancer cells.

**Figure 10:** Overexpressed miR-126-3p Inhibited Tumor Growth and Metastasis of Pancreatic Cancer (A) The effect of BMSCs-miR-126-3p mimic on the growth of the tumor detected by xenograft in nude mice. (B) Effect of BMSCs-miR-126-3p mimic on tumor volume detected by xenograft in nude mice. (C) Effect of BMSCs-miR-126-3p mimic on the quality of the tumor detected by xenograft in nude mice. (D) Expression of miR-126-3p and ADAM9 after BMSCs-miR-126-3p mimic treatment determined by qRT-PCR. (E and F) Protein expression of ADAM9, COX-2, and MMP-14 determined by western blot analysis (photograph of protein expression of ADAM9, COX-2, and MMP-14, E, and relative protein expression of ADAM9, COX-2, and MMP-14, F). *p < 0.05, compared with the BMSCs-miR-126-3p NC group. The data in the map were all measurement data and expressed by mean ± SD. (A) Data were analyzed by repeated-measurement variance of analysis. (C–E) Data were analyzed by independent sample t test for statistical analysis. n = 12. BMSC, human bone mesenchymal stem cell; COX-2, cyclooxygenase-2; miR-126-3p, microRNA-126-3p; MMP-14, matrix metalloproteinase-14; NC, negative control.

## Discussion

As the fourth main cause of cancer-related mortality, pancreatic cancer has had a survival rate of less than 5% for many decades due to few effective therapies.^3^ miRNAs have been highlighted because of their potential as cancer biomarkers and close association with the processes of tumorigenesis and various physiological and pathological developments including cell proliferation, differentiation, and apoptosis.^16^, ^22^ In our study, the specific mechanism by which miR-126-3p transferred via BMSC-derived exosomes influenced the biological function of pancreatic cancer was identified. The findings demonstrated that miR-126-3p shuttled by BMSC-derived exosome, by downregulating ADAM9, suppressed proliferation, invasion, and metastasis and promoted apoptosis in pancreatic cancer cells, thus acting as a potential biomarker for the treatment of pancreatic cancer.

Initially, miR-126-3p was noted to be poorly expressed, whereas ADAM9 was highly expressed in pancreatic cancer cell lines, with our results suggesting that miR-126-3p could directly inhibit the expression of ADAM9. Studies have indicated that miR-126-3p is poorly expressed in various tumors, including hepatocellular carcinoma, a finding which was consistent with the results of our study.^19^ The downregulation of miR-126-3p has also been flagged in cervical cancer tissues when compared with normal cervical tissues,^28^, ^29^, ^30^ whereas its level in cervical mucus was found to be increased among patients with cervical cancer.^31^ Furthermore, decreased miR-126 expression has been previously linked with pancreatic cancer.^24^, ^32^ Existing literature has suggested that ADAM9 is overexpressed during the progression of cancer in addition to indicating that silencing ADAM9 could promote both the radio-sensitivity and chemosensitivity of cancer cells to therapeutic drugs.^33^ Statistical evidence has demonstrated that pancreatic cancer cells exhibit a significantly higher level of ADAM9, which was also observed in the current study.^34^ Liu et al.^20^ concluded that miR-126 could suppress the expression of ADAM9 and act to further inhibit the growth of the ESCC through the epidermal growth factor receptor (EGFR)-AKT pathway. Various reports have pointed to the fact that pancreatic cancer cells exhibit downregulated levels of miR-126-3p and upregulated ADAM9, in addition to revealing that ADAM9 is a target gene of miR-126-3p, which acts to directly inhibit ADAM9.

Exosomes are membrane-enclosed small vesicles (30–100 nm) with endosomal origin that contain numerous molecular components including proteins, mRNAs, as well as miRNAs.^35^ Exosomes secreted by cells play a crucial role in correlating cells and transmitting information among tissues over long distances.^36^ BMSCs have been demonstrated to interact with tumor cells and participate in the progression of multiple tumors, including the processes of cell migration, invasion, and proliferation.^37^ More specifically, miR-31a-5p transferred by BMSC-derived exosomes has been shown to influence osteogenesis and osteoclastic differentiation.^38^ During the current study, a key observation was made indicating that BMSC-derived exosomes enriched miR-126-3p. Additionally, miR-126 enriched in exosomes from normal endothelial cells has been reported to contribute to suppressing cell growth and reducing the malignancy of non-small cell lung cancer cells.^39^ Studies have suggested that exosomes derived from BMSCs could alleviate liver injury of autoimmune hepatitis, which is correlated to the negative regulation of exosomal miR-233 on nucleotide-binding domain and leucine-rich repeat containing protein (NLR) pyrin domain containing 3.^40^

The abnormal expression of miRNAs has been widely associated with various human tumors and can be delivered to immune cells by exosomes secreted by tumors.^41^ Our results provided evidence demonstrating that miR-126-3p transferred by BMSC-derived exosomes could act to inhibit proliferation, migration, and invasion while promoting the apoptosis of pancreatic cancer cells via the downregulation of ADAM9. Hamada et al.^24^ asserted that upregulation of miR-126 in connection with the knockdown of ADAM9 leads to a reduction in cellular metastasis and invasion in pancreatic cancer, highlighting the crucial role of the miR-126/ADAM9 axis in inhibiting the invasive growth of pancreatic cancer cell lines. Moreover, silencing of ADAM9 has been shown to suppress proliferation and induce cell-cycle arrest in G1/G0 phase in prostate cancer cells.^33^ In our study, proliferation-related factors (Ki67 and VEGF) and invasion-related factors (COX-2 and MMP-14) were decreased with the overexpression of miR-126-3p. Ki67, a nuclear protein, could potentially serve as a marker during the processes of cell proliferation and cell growth, whereas VEGF has been highlighted as an important regulator in tumor angiogenesis.^42^ COX-2 and MMPs have been reported to influence inflammatory angiogenesis.^43^ In accordance with our study, studies have reported that miR-126 could target VEGF-A, whereas the expression of miR-126 has been shown to have a negative relationship with VEGF-A activity, as well as the expression of MMP-14 in cases of lung cancer.^44^, ^45^

In conclusion, the key findings of the present study present evidence indicating that miR-126-3p transferred by BMSCs secreted exosomes acts to suppress proliferation, migration, and invasion, while elevating the rate of apoptosis in pancreatic cancer cells by downregulating ADAM9 (Figure 11). The observations and data highlight the potential of miR-126-3p as a target for pancreatic cancer treatment. However, this study has its own shortcomings especially with small sample size. Further study concentrating on selection of two or more cell lines and selection of more animal experiments might increase the credibility and implication of the results.

**Figure 11:** miR-126-3p Transferred by BMSC-Derived Exosomes Entered Pancreatic Cancer Cells miR-126-3p can enter BMSC-derived exosomes and then be transferred to pancreatic cancer cells. In pancreatic cancer cells, miR-126-3p, by downregulating ADAM9 gene, decreases the expression of Ki67, VEGF, COX-2, and MMP-14, thus inhibiting proliferation, migration, and invasion and promoting apoptosis of pancreatic cancer cells. ADAM9, a disintegrin and metalloprotease-9; BMSC, bone marrow mesenchymal stem cell; COX-2, cyclooxygenase-2; miR-126-3p, microRNA-126-3p; MMP-14, matrix metalloproteinase-14; VEGF, vascular endothelial growth factor.

## Materials and Methods

### Ethics Statement

This study was approved by the Institutional Review Board and the Institutional Animal Care and Use Committee of School of Life Science, College of Health Sciences, Jiangsu Normal University. Written informed consents were obtained from all patients or guardians prior to their participation. All animal experiments were performed in strict adherence with the principle of using the smallest number of animals in order to complete the experiments. Extensive efforts were made to ensure the pain experienced by the animals during the experiments was minimal.

### Microarray Analysis

Through the retrieval of the GEO database (https://www.ncbi.nlm.nih.gov/geo/), four pancreatic cancer correlated gene chips (GEO: GSE16515, GSE32676, GSE71989, and GSE101448) and one miRNA chip (GEO: GSE28955) were retrieved (Table 1). The abnormal expressed genes in pancreatic cancer were screened from the four gene expression chips. Affy installation package in R language^46^ was employed in order to standardize the pretreatment of the chip expression data. The limma package^47^ was used for differential gene screening with |log2 FC| > 1.0, and *adj.P.Val* (corrected p value) < 0.05 was set as the threshold. Next, the expression thermal map of differential genes was constructed. The Calculate and draw custom Venn diagrams (http://bioinformatics.psb.ugent.be/webtools/Venn/) were used to compare the differential genes in four gene chips. The GEPIA database (http://gepia.cancer-pku.cn/)^48^ was employed to verify the expression of differential genes and analyze the correlation between gene expression and survival conditions. TargetScan (http://www.targetscan.org/vert_71/), miRSearch (http://www.exiqon.com/microrna-target-prediction), miRTarBase (http://mirtarbase.mbc.nctu.edu.tw/php/search.php), miRWalk (http://mirwalk.umm.uni-heidelberg.de/), and mirDIP (http://ophid.utoronto.ca/mirDIP/), five miRNA-mRNA relation prediction databases, were applied to predict the target miRNA of differentially expressed genes and compare predicted results of five miRNAs. The miRNA expression chip GEO: GSE28955 of pancreatic cancer was analyzed by R language using the same method of gene expression chip. Differentially expressed miRNAs in pancreatic cancer tissues were screened and compared with the target miRNAs of the differential genes.

**Table 1:** Information of Pancreatic Cancer Chip

Accession No.	Platform	Organism	Gene or miRNA	Sample
GEO: GSE16515	GPL570	*Homo sapiens*	gene	36 pancreatic cancer tumor samples and 16 normal samples
GEO: GSE32676	GPL570	*Homo sapiens*	gene	25 pancreatic cancer tumors and 7 non-malignant pancreas samples
GEO: GSE71989	GPL570	*Homo sapiens*	gene	8 normal pancreatic and 14 pancreatic ductal adenocarcinoma tissues
GEO: GSE101448	GPL10558	*Homo sapiens*	gene	18 with pancreatic tumor and 13 non-tumor pancreatic tissue samples
GEO: GSE28955	GPL6955	*Homo sapiens*	miRNA	16 pancreatic cancer cell lines and 4 normal pancreatic samples

### Cell Culture and Tissue Collection

Six pancreatic cancer cell lines, SW1990, Capan-1, AsPC-1, MIAPaCa-2, PANC-1, and PC-3, and human normal pancreatic cell line HPC-Y5 were purchased from Shanghai YanHui Biotechnical (Shanghai, China).

Specimens from 28 patients with pancreatic cancer and 32 patients with pancreatitis who had undergone surgical resection procedures at the School of Life Science, College of Health Sciences, Jiangsu Normal University from January 2018 to May 2018 were recruited for the purposes of the study. Five pancreatic cancer tissues and five pancreatitis tissues were promptly excised using sharp knives within a period of 5 min after the specimens had been removed from the patients. All patients enrolled into the study were yet to be administered chemotherapy, radiotherapy, or immunotherapy prior to surgery, in addition to being pathologically diagnosed postoperatively independently by two pathologists. Tissue samples were obtained and immediately preserved in liquid nitrogen and stored at −70°C.

### Plasmids and Lentivirus Transfection

Pancreatic cancer cells were inoculated into six-well plates (2 × 10^5^ cells/well) 1 day prior to transfection. Transfection was performed when cell confluence was confirmed to have reached 60%–80%. The cells were transfected with miR-126-3p/NC mimic, miR-126-3p/NC inhibitor, and shADAM9/NC plasmids using Lipofectamine 2000 (Carlsbad, CA, USA) in accordance with the instructions provided. In an attempt to reduce toxicity, the transfection complex was replaced with fresh medium after 6 h had elapsed. The cells were analyzed and further examined 48 h after transfection.

Lentivirus packaging was performed in a 60-mm culture vessel that contains 1 mm pMD2G, 3 μg psPAX2, and 4 μg Prutou3-mChely/LuxIFEase/mimic NC/miR-126-3p using the transient co-transfection system of HEK293T cells. 24 h after transfection, supernatant was collected, following the addition of a fresh medium for the second supernatant collection after 24 h. The two aforementioned supernatants were then mixed for target cell infection purposes. Lentivirus-transfected BMSCs were cultured overnight in 24-well plates at a density of 5 × 10^4^ cells/well. Medium containing 500 μL lentivirus supernatant, 500 μL fresh culture medium, and 8 μg polyacrylamide (Sigma, St. Louis, MO, USA) was used to facilitate the uptake of virus particles. Then the plate was centrifuged (7,890 × *g*) at 37°C, then permitted to react for 1 h and replaced with fresh medium. The cells were screened by 7 g/mL rodenticidin postinfection, and the DsRed fluorescence was observed under the fluorescence microscope (MICHE) 7 days later.

### Dual-Luciferase Reporter Gene Assay

Bioinformatics database (microRNA.org; http://www.microrna.org/microrna/home.do) was used to provide information predicting whether ADAM9 was indeed a target gene of miR-126-3p. Human embryo kidney HEK293T cells were cultured in DMEM containing 10% fetal bovine serum (FBS) at 37°C with 5% CO_2_. The cDNA fragment in ADAM9 3′UTR containing miR-126-3p binding sites was inserted into pmirGLO vector. The cDNA fragments of ADAM9 3′ UTR with binding site mutation were inserted into pmirGLO vector. The recombinant vector of pmirGLO-ADAM9 or pmirGLO-mutADAM9 was co-transfected with miR-126-3p mimic (miR-126-3p overexpression sequence) or miR-NC (NC sequence) into HEK293T cells by liposome transfection, respectively. Subsequently, the cells were then cultured for 48 h, collected, and lysed. A total volume of 100 μL lysate supernatant was added with 100 μL renilla luciferase detection fluid in order to determine the renilla luciferase activity. In addition, 100 μL lysate supernatant was mixed with 100 μL firefly luciferase detection reagent in order to detect the firefly luciferase activity. The renilla luciferase and firefly luciferase activities were detected by the multifunctional enzyme analyzer SpectraMaxM5 for 10 s at 2-s interval.

### 5-Ethynyl-2′-Deoxyuridine

Cells exhibiting logarithmic growth were inoculated into 96-well plates at a density of 4 × 10^3^ to 1 × 10^5^ cells/well and cultured until to normal cell development stage. The cell culture medium was used to dilute 5-ethynyl-2′-deoxyuridine (EdU) solution at a ratio of 1000:1, and 50 μM EdU culture medium was prepared accordingly. The cells were incubated with 100 μL EdU (50 μM) culture medium for 2 h and then abandoned. The cells were fixed with 50 μL cell fixative solution (PBS containing 4% paraformaldehyde) for 30 min; then the fixative solution was discarded. After 50 μL (2 mg/mL) glycine was added, cells were incubated in the decolorized shaker for 5 min, after which the glycine solution was discarded. The cells were then incubated for 10 min in a decolorized shaker with 100 μL infiltrator (PBS containing 0.5% Triton X-100). Next, 100 μL 1× Apollo staining reaction liquid was added to the cells and incubated in a decolorized shaker under conditions void of light for 30 min followed by the removal of the reactive liquid. The cells were then washed with 100 μL infiltrator (PBS containing 0.5% Triton X-100) in decolorized shaker two to three times, each time for 10 min, followed by the removal of infiltrator. Reagent F was diluted by deionized water at a ratio of 100:1 to prepared moderate 1× Hoechst 33342 staining reaction liquid, which was preserved in dark conditions void of sunlight. The cells were added with 100 μL 1× Hoechst 33342 and incubated in a decolorized shaker avoiding exposure to light for 30 min, followed by the removal of reactive liquid.

### Transwell Assay

Detection of cell migration was performed as follows: in the event that cell confluence reached 80%, the third-generation cells were starved in the serum-free DMEM culture medium for 24 h. Serum-free DMEM culture medium was added to the bottom of the Transwell chambers (Corning, NY, USA) and placed at 37°C for 1 h. After digestion, the cells were resuspended with serum-free DMEM, counted, and diluted to 3 × 10^5^ cells/mL, of which 100 μL was added to the apical chamber. At the same time, 600 μL DMEM with 10% serum (serum was taken as chemokines) was added into the basolateral chamber and incubated for 24 h in accordance with the instructions of the Transwell chamber. The cells from the apical chamber were soaked in precooled methanol for 30 min, then fixed and transferred into the basolateral chamber. Subsequently, the cells were stained with 0.1% crystalline violet solution for 10 min. The cells were then photographed and counted under an inverted microscope (Olympus, Tokyo, Japan) with six visual fields selected.

Detection of cell invasion was performed as follows: Matrigel preserved at −20°C was melted at 4°C and diluted using serum-free DMEM with the remaining procedures performed in an identical fashion to the steps used for cell migration.

### Flow Cytometry

Annexin V-FITC and/or propidium iodide (PI) double standard staining was employed to detect cell apoptosis. The cells were collected 48 h after transfection with the concentration adjusted to 1 × 10^6^ cells/mL. Cells were fixed overnight with 70% precooled ethanol solution at 4°C. 100 μL cell suspension (no less than 10^6^ cells/mL) was centrifuged. The cells were subsequently resuspended in 200 μL binding buffer and gently mixed with 10 μL Annexin V-FITC and 5 μL PI under conditions void of light for 15 min, followed by the addition of 300 μL binding buffer. Cell apoptosis was detected using flow cytometry at an excitation wavelength of 488 nm.

### Isolation and Identification of BMSCs

Under sterile conditions, 10 mL bone marrow was extracted from the femoral shaft fracture end with a 20-mL syringe (containing 2,000 IU heparin) and mixed with heparin quickly. The bone marrow was centrifuged in a centrifuge tube at 258 × *g* for 10 min in order to remove the upper adipose tissue, followed by three washes with DMEM, and resuspended using 15 mL medium. Bone marrow was centrifuged in a centrifuge tube containing the same volume of Ficoll-Paque PLUS lymphocyte separation fluid at 716 × *g* for 20 min. Nucleated cells were noted to be located predominately in the boundary and upper liquids, while most of the erythrocytes had precipitated to the bottom. The nuclear cells were withdrawn from the interface with a straw, centrifuged at 179 × *g* for 8 min, after which the supernatant was discarded. Next, 5 mL cell culture medium was added to make nuclear cells evenly spread. The cell suspension (10 μL) was evenly mixed with 490 μL PBS. After that, 10 μL of mixture was obtained and counted under the microscope. The cells were inoculated in a culture bottle (1 × 10^5^ cells/bottle) and incubated with 5 mL low-glucose DMEM culture medium at 37°C with 5% CO_2_ and saturated humidity. After 24 h, BMSCs began to adhere to the wall, and half of the medium was replaced to remove non-adherent cells. The medium was replaced every 2–3 days, during which a small amount of hematopoietic stem cells, as well as the red blood cell suspension that failed to be removed by means of centrifugation, along with the other non-adherent mixed cells, was removed in a progressive manner. Cell adhesion and growth were observed using an inverted phase-contrast microscope. When the monolayer adherent cells grew to 80%–90% confluence at days *in vitro* (DIV) 10–14, the cells were treated with 0.25% trypsin and sub-cultured at ratio of 1:2–1:3. Flow cytometer was used to detect surface markers CD29, CD34, CD44, CD45, CD71, and HLA-DR of BMSCs. The adipogenic and osteogenic differentiation of BMSCs was identified according to the ability of inducing differentiation *in vitro*, and the formation of lipid droplets was observed by oil red O staining under an inverted microscope. The calcium deposits of osteoblast differentiation were observed through the application of alizarin red staining 4 weeks after osteoblast induction and differentiation.

### Exosomes Extraction

The exosomes in serum were removed by means of ultracentrifugation of FBS at 100,000 × *g* for 8 h. When BMSCs’ confluence reached around 80%, the supernatant was removed. BMSCS were cultured in 10% exosome-free FBS at 37°C in a CO_2_ incubator for 48 h. The collected supernatant was centrifuged in a gradual manner at varying speeds according to the following steps: 300 × *g* for 10 min at 4°C with the removal of the precipitation, at 2,000 × *g* for 15 min at 4°C with the precipitation removed, at 5,000 × *g* for 15 min at 4°C with the precipitation removed, and at 12,000 × *g* for 30 min at 4°C following the collection of the precipitation. The supernatant was subsequently centrifuged at 12,000 × *g* for 70 min at 4°C with the precipitation collected. The supernatant following centrifugation was centrifuged at overspeed for 70 min at 100,000 × *g* at 4°C, after which the precipitation was collected, followed by centrifugation for 70 min at 100,000 × *g* at 4°C with the precipitation collected.

### Nanoparticles Tracking Analysis

20 μg of exosomes was dissolved in 1 mL PBS and vortexed for 1 min in order to ensure a uniform distribution. NanoSight nanoparticle tracking analyzer (Malvern Panalytical, Worcestershire, UK) was employed in order to directly determine the size distribution.

### Transmission Electron Microscopy Observation

The prepared exosomes were promptly fixed in 4% glutaraldehyde for fixation purposes for 2 h under 4°C conditions, fixed with 1% osmium tetroxide for 2 h, and dehydrated using conventional gradient ethanol and acetone. The exosomes were immersed, embedded, and polymerized with ethoxyline resin to prepare slices at a thickness of 0.5 μm. After positioning under a light microscope, ultrathin slices with a thickness of 60 μm were prepared, stained with uranium acetate and lead citron citrate, and observed under an electron microscope.

### Acetylcholinesterase Activity Assay

Exosomes extracted using multistep ultracentrifugation were diluted with PBS to 110 μL. Cells in each well in the 96-well plate were added with a solution containing PBS and 5,5′-dithiobis-2-nitrobenzoic acid (DTNB) solution (0.1 mmol/L) with equal volume (37.5 μL); then the acetylcholine solution of sulfur iodide (1.25 mmol/L) was added to a final volume of 300 μL. After 30 min, the optical density (OD) values of each well were detected using a microplate reader at a wavelength of 412 nm.

### Co-culture of Pancreatic Cancer Cells and BMSCs

The pancreatic cancer cell lines PANC-1 and BMSCs were attached with trypsin, centrifuged at 1,000 × *g* for 5 min, and resuspended with 3 mL DMEM culture medium. Next, 1 mL suspension was diluted 20 times more. The diluted cell suspension was fully mixed, and 10 μL resuspension was counted under the cell count plate. Finally, PANC-1 and BMSCs, at the ratio of 3:1, were spread to a diameter of 0.4 μm co-culture chamber. In the co-culture chamber, BMSCs (about 0.4 × 10^5^) were placed into the basolateral chamber, whereas PANA-1 cells (about 1.2 × 10^5^) were placed into the apical chamber, with the co-culture chamber placed in the six-well plate. The PANC-1 cells in the apical chamber were cultured with DMEM containing 10% serum, and BMSCs cells in the basolateral chamber were cultured in DMEM culture medium containing 15% serum for 4–5 days with the liquid and medium in both apical and basolateral chambers changed every 1–2 days. After co-culturing, the apical chamber was withdrawn and the cells were used for subsequent experiments.

### Confocal Fluorescence Microscopy

BMSCs transfected with miR-126-3p-Cy3 (GenePharma, Shanghai, China) carrying red fluorescent markers were co-cultured with pancreatic cancer cells transfected with pCDNA3.1-GFP. The uptake of the exosomes by pancreatic cancer cells was observed under a confocal fluorescence microscope after 6, 24, and 48 h of co-culture, respectively. After 2 days of co-culture, two cell lines were separated by flow cytometry.

### RNA Isolation and Quantitation

Total RNA from the cells was extracted by TRIzol (Invitrogen, Carlsbad, CA, USA). After determination of RNA concentration using NanoDrop2000 (Thermo Fisher Scientific, Waltham, MA, USA), 1 μg total RNA was reversely transcribed into cDNA using the PrimeScript RT reagent kit with gDNA Eraser Kit (Takara Bio, Otsu, Shiga, Japan). Following the addition of 5 × *g* DNA Eraser Buffer and gDNA Eraser, DNA removal was conducted at 42°C for 2 min. Next, RNA was reversely transcribed into cDNA. qRT-PCR was performed using a ABI7500 quantitative PCR instrument (Thermo Fisher Scientific, Waltham, MA, USA) with the SYBR PremixExTaq (TliRNaseHPlus) kits (Takara Bio, Otsu, Shiga, Japan). U6 was regarded as the internal reference for miR-126-3p, whereas glyceraldehyde-3-phosphate dehydrogenase (GAPDH) was considered the internal reference for the others. The 2^−ΔΔCt^ method was applied to express the ratio of expression of the target gene in the experimental group and the reference group. The formula was as follows: ΔΔCT (comparative threshold cycle) = Ct_the experimental group_ − Ct_the NC group_, ΔCT = Ct_gene_ − Ct_internal control_.^49^ The cycle threshold (Ct) was considered to be reflective of the number of amplification cycles when the real-time fluorescence intensity reached the set threshold, and the amplification was logarithmic. The primers used in the reaction are displayed in Table 2. The primers used were provided by Gemma Pharmaceutical Technology (Shanghai, China).

**Table 2:** Primer Sequence for qRT-PCR

Gene	Sequence	
miR-126-3p	F	5′-GCTGGCGACGGGACATTA-3′
	R	5′-CGCATTATATACTCACGGAAGG-3′
U6	F	5′-CTCGCTTCGGCAGCACA-3′
	R	5′-AACGCTTCACGAATTTGCGT-3′
ADAM9	F	5′-GCTGTCTTGCCACAGACCC GGTATGTGGAG-3′
	R	5′-TGGAATATTAAGAAGGCAGTT TCCTCCTTT-3′
GAPDH	F	5′-CCCACTCCTCCACCTTTGAC-3′
	R	5′-ATGAGGTCCACCACCCTGTT-3′

ADAM9, a disintegrin and a metalloproteinase-9; F, forward; GAPDH, glyceraldehyde-3-phosphate dehydrogenase; miR-126-3p, microRNA-126-3p; R, reverse.

### Western Blot Analysis

The total protein was extracted and the protein concentration was assayed by bicinchoninic acid (BCA) kit (Thermo Fisher Scientific, Waltham, MA, USA). After polyacrylamide gel electrophoresis for 35 min at constant voltage 80 V and 45 min at 120 V, total protein (30 μg) was transferred to polyvinylidene fluoride membrane (Amersham Biosciences, Boston, MA, USA), sealed for 1 h with 5% skimmed milk powder, followed by the removal of the sealing liquid. After that, the membrane was incubated with rabbit monoclonal antibody to CD63 (1:1,000, ab134045), rabbit polyclonal antibodies to Hsp70 (1:1,000, ab79852), Ki67 (1:5,000, ab15580), VEGF (1:1,000, ab2349), MMP-14 (1:5,000, ab38971), COX-2 (1:1,000, ab15191), and GAPDH rabbit antibody (1:5,000, ab181602) overnight at 4°C. All the aforementioned antibodies were purchased from Abcam (Cambridge, UK). The membrane was washed three times with PBS-Tween 20 (PBST) (containing 0.1% Tween-20 PBS buffer), 10 min for each. After the addition of horseradish peroxidase-labeled goat anti-rabbit secondary antibody (1:10,000; Jackson ImmunoResearch Laboratories, West Grove, PA, USA), the membrane was incubated for 1 h, scanned, and developed under an optical luminescence instrument (General Electric Company, Boston, MA, USA). ImageProPlus 6.0 (MediaCybernetics, MD, USA) software was used for protein band scanning and analyzing the relative protein expression. Three parallel experiments were repeated.

### Xenograft in Nude Mice

Male BALB/c nude mice (4–6 weeks, 20–25 g) were obtained from the experimental animal center (Chinese Academy of Sciences, Shanghai, China) were fed at a constant temperature (25°C–27°C) and constant humidity (45%–50%). The nude mice were randomly classified into two groups with 12 mice placed in each group. After anesthesia, the mice were inoculated with cells. The pancreatic cancer cells exhibiting logarithmic growth were resuspended in 50% Matrigel (BD Biosciences, Bedford, MA, USA) with the cell concentration adjusted to 2 × 10^6^ cells/mL, and 0.2-mL single-cell suspension (4 × 10^5^ cells) was subcutaneously injected into left subaxillary skin of each nude mouse, respectively. After the tumor had grown to approximately 100 mm^3^, the mice were injected with lentivirus-packaged BMSCs. BMSCs were transiently transfected with miR-NC or miR-126-3p. After the BALB/c nude mice were injected with lentivirus-packaged BMSCs, the tumor volume (mm^3^) was calculated using the formula: (L × W^2^)/2, in which L was the tumor length unit and W was the width unit of the tumor. After seven rounds of treatment, the nude mice were euthanized by means of anesthesia. The tumors were collected and weighed, with certain tumor tissues reserved for qRT-PCR and western blot analysis.

### Statistical Analysis

Statistical analysis was conducted using SPSS 21.0 (IBM, Armonk, NY, USA) software. Normal distribution test and homogeneity of variance were conducted. Data displaying normal distribution were expressed as mean ± SD. The data of patients with pancreatic cancer and pancreatitis were compared using an independent sample t test. Data failing to conform to homogeneity of variance were corrected by Welch’s t test. One-way ANOVA was used for comparison among multiple groups, while data between two groups were compared by Tukey for backing test. All the data with skew distribution were tested by nonparametric tests. Data at different times points were analyzed by repeated-measurement ANOVA. p < 0.05 was considered to be indicative of statistical significance.

## Author Contributions

D.-M.W, J.L., G.-Q.C., and Y.-L.Z. designed the study. X.W., X.-R.H., S.W., Y.-J.W., and M.S. collated the data, and designed and developed the database. S.-H.F., Z.-F.Z., Q.S., M.-Q.L., and B.H. carried out data analyses and produced the initial draft of the manuscript. D.-M.W., J.L., G.-Q.C., and Y.-L.Z. contributed to drafting the manuscript. All authors have read and approved the final submitted manuscript.

## Conflicts of Interest

The authors declare no competing interests.

## Supplemental Information

Table S1. The Raw Data for the Experimental Statistical Analysis of Figure 1A

Table S2. The Raw Data for the Experimental Statistical Analysis of Figure 1H

Table S3. The Raw Data for the Experimental Statistical Analysis of Figures 1D, 1E, and 1I

## References

[1] Waddell N., Pajic M., Patch A.M., Chang D.K., Kassahn K.S., Bailey P., Johns A.L., Miller D., Nones K., Quek K., Australian Pancreatic Cancer Genome Initiative (2015). Whole genomes redefine the mutational landscape of pancreatic cancer. Nature.

[2] Jacobetz M.A., Chan D.S., Neesse A., Bapiro T.E., Cook N., Frese K.K., Feig C., Nakagawa T., Caldwell M.E., Zecchini H.I. (2013). Hyaluronan impairs vascular function and drug delivery in a mouse model of pancreatic cancer. Gut.

[3] Biankin A.V., Waddell N., Kassahn K.S., Gingras M.C., Muthuswamy L.B., Johns A.L., Miller D.K., Wilson P.J., Patch A.M., Wu J., Australian Pancreatic Cancer Genome Initiative (2012). Pancreatic cancer genomes reveal aberrations in axon guidance pathway genes. Nature.

[4] Giovannetti E., Funel N., Peters G.J., Del Chiaro M., Erozenci L.A., Vasile E., Leon L.G., Pollina L.E., Groen A., Falcone A. (2010). MicroRNA-21 in pancreatic cancer: correlation with clinical outcome and pharmacologic aspects underlying its role in the modulation of gemcitabine activity. Cancer Res..

[5] Ali S., Saleh H., Sethi S., Sarkar F.H., Philip P.A. (2012). MicroRNA profiling of diagnostic needle aspirates from patients with pancreatic cancer. Br. J. Cancer.

[6] Wakitani S., Okabe T., Horibe S., Mitsuoka T., Saito M., Koyama T., Nawata M., Tensho K., Kato H., Uematsu K. (2011). Safety of autologous bone marrow-derived mesenchymal stem cell transplantation for cartilage repair in 41 patients with 45 joints followed for up to 11 years and 5 months. J. Tissue Eng. Regen. Med..

[7] Liu X., Duan B., Cheng Z., Jia X., Mao L., Fu H., Che Y., Ou L., Liu L., Kong D. (2011). SDF-1/CXCR4 axis modulates bone marrow mesenchymal stem cell apoptosis, migration and cytokine secretion. Protein Cell.

[8] Mathew E., Brannon A.L., Del Vecchio A., Garcia P.E., Penny M.K., Kane K.T., Vinta A., Buckanovich R.J., di Magliano M.P. (2016). Mesenchymal Stem Cells Promote Pancreatic Tumor Growth by Inducing Alternative Polarization of Macrophages. Neoplasia.

[9] Wu X.B., Liu Y., Wang G.H., Xu X., Cai Y., Wang H.Y., Li Y.Q., Meng H.F., Dai F., Jin J.D. (2016). Mesenchymal stem cells promote colorectal cancer progression through AMPK/mTOR-mediated NF-κB activation. Sci. Rep..

[10] Yan X., Zhang D., Wu W., Wu S., Qian J., Hao Y., Yan F., Zhu P., Wu J., Huang G. (2017). Mesenchymal Stem Cells Promote Hepatocarcinogenesis via lncRNA-MUF Interaction with ANXA2 and miR-34a. Cancer Res..

[11] Choi M.R., Kim H.Y., Park J.Y., Lee T.Y., Baik C.S., Chai Y.G., Jung K.H., Park K.S., Roh W., Kim K.S., Kim S.H. (2010). Selection of optimal passage of bone marrow-derived mesenchymal stem cells for stem cell therapy in patients with amyotrophic lateral sclerosis. Neurosci. Lett..

[12] Sun Y.P., Zhang B.L., Duan J.W., Wu H.H., Wang B.Q., Yu Z.P., Yang W.J., Shan Y.F., Zhou M.T., Zhang Q.Y. (2014). Effect of NK4 transduction in bone marrow-derived mesenchymal stem cells on biological characteristics of pancreatic cancer cells. Int. J. Mol. Sci..

[13] Marote A., Teixeira F.G., Mendes-Pinheiro B., Salgado A.J. (2016). MSCs-Derived Exosomes: Cell-Secreted Nanovesicles with Regenerative Potential. Front. Pharmacol..

[14] Yu B., Shao H., Su C., Jiang Y., Chen X., Bai L., Zhang Y., Li Q., Zhang X., Li X. (2016). Exosomes derived from MSCs ameliorate retinal laser injury partially by inhibition of MCP-1. Sci. Rep..

[15] Ohno S., Takanashi M., Sudo K., Ueda S., Ishikawa A., Matsuyama N., Fujita K., Mizutani T., Ohgi T., Ochiya T. (2013). Systemically injected exosomes targeted to EGFR deliver antitumor microRNA to breast cancer cells. Mol. Ther..

[16] Shibayama Y., Kondo T., Ohya H., Fujisawa S., Teshima T., Iseki K. (2015). Upregulation of microRNA-126-5p is associated with drug resistance to cytarabine and poor prognosis in AML patients. Oncol. Rep..

[17] Xie V.K., Li Z., Yan Y., Jia Z., Zuo X., Ju Z., Wang J., Du J., Xie D., Xie K., Wei D. (2017). DNA-Methyltransferase 1 Induces Dedifferentiation of Pancreatic Cancer Cells through Silencing of Krüppel-Like Factor 4 Expression. Clin. Cancer Res..

[18] Cui W., Li Q., Feng L., Ding W. (2011). MiR-126-3p regulates progesterone receptors and involves development and lactation of mouse mammary gland. Mol. Cell. Biochem..

[19] Du C., Lv Z., Cao L., Ding C., Gyabaah O.A., Xie H., Zhou L., Wu J., Zheng S. (2014). MiR-126-3p suppresses tumor metastasis and angiogenesis of hepatocellular carcinoma by targeting LRP6 and PIK3R2. J. Transl. Med..

[20] Liu R., Gu J., Jiang P., Zheng Y., Liu X., Jiang X., Huang E., Xiong S., Xu F., Liu G. (2015). DNMT1-microRNA126 epigenetic circuit contributes to esophageal squamous cell carcinoma growth via ADAM9-EGFR-AKT signaling. Clin. Cancer Res..

[21] Cao Z., Liu C., Xu J., You L., Wang C., Lou W., Sun B., Miao Y., Liu X., Wang X. (2016). Plasma microRNA panels to diagnose pancreatic cancer: Results from a multicenter study. Oncotarget.

[22] Xiong Y., Kotian S., Zeiger M.A., Zhang L., Kebebew E. (2015). miR-126-3p Inhibits Thyroid Cancer Cell Growth and Metastasis, and Is Associated with Aggressive Thyroid Cancer. PLoS ONE.

[23] Xu Q., Liu X., Cai Y., Yu Y., Chen W. (2010). RNAi-mediated ADAM9 gene silencing inhibits metastasis of adenoid cystic carcinoma cells. Tumour Biol..

[24] Hamada S., Satoh K., Fujibuchi W., Hirota M., Kanno A., Unno J., Masamune A., Kikuta K., Kume K., Shimosegawa T. (2012). MiR-126 acts as a tumor suppressor in pancreatic cancer cells via the regulation of ADAM9. Mol. Cancer Res..

[25] Bai C., Chen S., Gao Y., Shan Z., Guan W., Ma Y. (2015). Multi-lineage potential research of bone marrow mesenchymal stem cells from Bama miniature pig. J. Exp. Zoolog. B Mol. Dev. Evol..

[26] Wisniewski D., Affer M., Willshire J., Clarkson B. (2011). Further phenotypic characterization of the primitive lineage- CD34+CD38-CD90+CD45RA- hematopoietic stem cell/progenitor cell sub-population isolated from cord blood, mobilized peripheral blood and patients with chronic myelogenous leukemia. Blood Cancer J..

[27] Bergholtz B.O., Thoresen A.B., Thorsby E. (1980). HLA-D/DR restriction of macrophage-dependent antigen activation of immune T lymphocytes: cross-reacting allogeneic HLA-D/DR may partly substitute for self HLA-D/DR. Scand. J. Immunol..

[28] Shan G., Moonie S., Shen J. (2016). Sample size calculation based on efficient unconditional tests for clinical trials with historical controls. J. Biopharm. Stat..

[29] Huang T.H., Chu T.Y. (2014). Repression of miR-126 and upregulation of adrenomedullin in the stromal endothelium by cancer-stromal cross talks confers angiogenesis of cervical cancer. Oncogene.

[30] Wang X., Tang S., Le S.Y., Lu R., Rader J.S., Meyers C., Zheng Z.M. (2008). Aberrant expression of oncogenic and tumor-suppressive microRNAs in cervical cancer is required for cancer cell growth. PLoS ONE.

[31] Kawai S., Fujii T., Kukimoto I., Yamada H., Yamamoto N., Kuroda M., Otani S., Ichikawa R., Nishio E., Torii Y., Iwata A. (2018). Identification of miRNAs in cervical mucus as a novel diagnostic marker for cervical neoplasia. Sci. Rep..

[32] Frampton A.E., Krell J., Jacob J., Stebbing J., Castellano L., Jiao L.R. (2012). Loss of miR-126 is crucial to pancreatic cancer progression. Expert Rev. Anticancer Ther..

[33] Liu C.M., Hsieh C.L., He Y.C., Lo S.J., Liang J.A., Hsieh T.F., Josson S., Chung L.W., Hung M.C., Sung S.Y. (2013). In vivo targeting of ADAM9 gene expression using lentivirus-delivered shRNA suppresses prostate cancer growth by regulating REG4 dependent cell cycle progression. PLoS ONE.

[34] Yamada D., Ohuchida K., Mizumoto K., Ohhashi S., Yu J., Egami T., Fujita H., Nagai E., Tanaka M. (2007). Increased expression of ADAM 9 and ADAM 15 mRNA in pancreatic cancer. Anticancer Res..

[35] Yang Y., Ye Y., Su X., He J., Bai W., He X. (2017). MSCs-Derived Exosomes and Neuroinflammation, Neurogenesis and Therapy of Traumatic Brain Injury. Front. Cell. Neurosci..

[36] Xia Q., Li X., Zhou H., Zheng L., Shi J. (2018). S100A11 protects against neuronal cell apoptosis induced by cerebral ischemia via inhibiting the nuclear translocation of annexin A1. Cell Death Dis..

[37] Wang Y., Shao S., Luo M., Huang S., Feng L., Yuan N., Wu F., Dang C., Zhao X. (2017). Effects of rat bone marrow-derived mesenchymal stem cells on breast cancer cells with differing hormone receptor status. Oncol. Lett..

[38] Xu R., Shen X., Si Y., Fu Y., Zhu W., Xiao T., Fu Z., Zhang P., Cheng J., Jiang H. (2018). MicroRNA-31a-5p from aging BMSCs links bone formation and resorption in the aged bone marrow microenvironment. Aging Cell.

[39] Grimolizzi F., Monaco F., Leoni F., Bracci M., Staffolani S., Bersaglieri C., Gaetani S., Valentino M., Amati M., Rubini C. (2017). Exosomal miR-126 as a circulating biomarker in non-small-cell lung cancer regulating cancer progression. Sci. Rep..

[40] Chen L., Lu F.B., Chen D.Z., Wu J.L., Hu E.D., Xu L.M., Zheng M.H., Li H., Huang Y., Jin X.Y. (2018). BMSCs-derived miR-223-containing exosomes contribute to liver protection in experimental autoimmune hepatitis. Mol. Immunol..

[41] Zhou M., Chen J., Zhou L., Chen W., Ding G., Cao L. (2014). Pancreatic cancer derived exosomes regulate the expression of TLR4 in dendritic cells via miR-203. Cell. Immunol..

[42] Chen J.X., Deng N., Chen X., Chen L.W., Qiu S.P., Li X.F., Li J.P. (2012). A novel molecular grading model: combination of Ki67 and VEGF in predicting tumor recurrence and progression in non-invasive urothelial bladder cancer. Asian Pac. J. Cancer Prev..

[43] Scoditti E., Calabriso N., Massaro M., Pellegrino M., Storelli C., Martines G., De Caterina R., Carluccio M.A. (2012). Mediterranean diet polyphenols reduce inflammatory angiogenesis through MMP-9 and COX-2 inhibition in human vascular endothelial cells: a potentially protective mechanism in atherosclerotic vascular disease and cancer. Arch. Biochem. Biophys..

[44] Sasahira T., Kurihara M., Bhawal U.K., Ueda N., Shimomoto T., Yamamoto K., Kirita T., Kuniyasu H. (2012). Downregulation of miR-126 induces angiogenesis and lymphangiogenesis by activation of VEGF-A in oral cancer. Br. J. Cancer.

[45] Xu M., Wang Y.Z. (2013). miR-133a suppresses cell proliferation, migration and invasion in human lung cancer by targeting MMP-14. Oncol. Rep..

[46] Gautier L., Cope L., Bolstad B.M., Irizarry R.A. (2004). affy—analysis of Affymetrix GeneChip data at the probe level. Bioinformatics.

[47] Smyth G.K. (2004). Linear models and empirical bayes methods for assessing differential expression in microarray experiments. Stat. Appl. Genet. Mol. Biol..

[48] Tang Z., Li C., Kang B., Gao G., Li C., Zhang Z. (2017). GEPIA: a web server for cancer and normal gene expression profiling and interactive analyses. Nucleic Acids Res..

[49] Livak K.J., Schmittgen T.D. (2001). Analysis of relative gene expression data using real-time quantitative PCR and the 2(-Delta Delta C(T)) Method. Methods.

